# TMEM60 Promotes the Proliferation and Migration and Inhibits the Apoptosis of Glioma through Modulating AKT Signaling

**DOI:** 10.1155/2022/9913700

**Published:** 2022-01-03

**Authors:** Jingwen Wu, Xinghua Tang, Xuejuan Yu, Xiaoli Zhang, Wenjun Yang, Ashima Seth, Qiuan Yang

**Affiliations:** ^1^Department of Radiation Oncology, Qilu Hospital, Cheeloo College of Medicine, Shandong University, Jinan, China; ^2^Master of Healthcare Administration at Price School of Public Policy, University of Southern California, Los Angeles, CA, USA

## Abstract

Glioma is a highly fatal malignancy with aggressive proliferation, migration, and invasion metastasis due to aberrant genetic regulation. This work aimed to determine the function of transmembrane protein 60 (TMEM60) during glioma development. The level of TMEM60 in glioma tissues and normal tissues and its correlation with glioma prognosis were checked in The Cancer Genome Atlas (TCGA) database. The levels of TMEM60 in glioma cell lines and normal astrocytes were determined by quantitative real-time PCR and western blotting assay. TMEM60 knockdown and overexpression were conducted, followed by detection of cell viability, migration, invasion, and apoptosis. CCK-8 and colony formation assay were adopted to detect cell viability proliferation. Transwell assay was performed to measure cell migration and invasion. Cell apoptosis was evaluated by flow cytometry. The alternation of key proteins in the PI3K/Akt signaling pathway was measured by western blotting. TMEM60 expression was significantly higher in glioma tissues than that in the healthy control and was correlated with poor overall survival of patients. The protein and mRNA levels of TMEM60 were both elevated in glioma cell lines in comparison with the normal cell lines. Elevated level of TMEM60 led to enhanced proliferation, migration, and invasion and suppressed cell apoptosis. TMEM60 promoted the activation of PI3K/Akt signaling. Our data suggested that TMEM60 plays an oncogenic role in glioma progression via activating the PI3K/Akt signaling pathway.

## 1. Introduction

Glioma is the most commonly occurring brain malignancy in adults, exhibiting highly aggressive feature and grave prognosis [1–3]. Numerous studies have disclosed that the progression of glioma is closely correlated with abnormal metabolism, vascular endothelial proliferation, and suppressed immune response [4–7]. Large-scale genome analysis and accumulating studies on molecular mechanisms have presented multiple oncogenes that contribute to glioma onset, such as Notch, platelet-derived growth factor receptor alpha (PDGFRA), and epithelial growth factor receptor (EGFR) [8–12]. For example, Notch signaling participates in the regulation of glioma cell stemness and promotes self-renewal of glioma cells [13–15]. Genomic sequencing unraveled the alteration of the EGFR gene in over 50% of glioma [8, 16].

Over the past decades, the developed therapeutic manners including surgical operation and chemo- and radiotherapy have successfully achieved partial remission in glioma patients, yet there still exist some patients who show slight response, and the 5-year relative survival is only 5% [9, 10, 17]. Therefore, it is urgent to decipher the mechanisms underlying the pathogenesis of glioma and develop safe and efficient therapeutic strategies. The phosphatidylinositol 3-kinases (PI3Ks)/Akt signaling pathway is a central regulator of signaling transduction during biological processes of cancer cells, such as viability, metastasis, metabolism, and angiogenesis [18–20]. The PI3K/Akt pathway could be activated by receptor tyrosine kinases (RTKs) or G protein-coupled receptors (GPCRs), during which the PI3K activates PIP3 to anchor Akt to cell membranes. The Akt is then phosphorylated activated by mTOR at Thr308 and Ser473 residues [21–23]. Previous studies have reported the important function of PI3K/Akt signaling in glioma and its potential as therapeutic targets [24–26].

In this present work, we, for the first time, confirmed the elevated expression of transmembrane protein 60 (TMEM60) in glioma tissue samples and cell lines. We evaluated cell viability, migration, invasion, and apoptosis after knockdown or ectopic expression of TMEM60 and determined the changes on the PI3K/Akt pathway. Our basic experimental findings provided novel evidences to uncover the TMEM60/PI3K/Akt signaling in glioma and supplied a notable perception concerning the regulatory axis in glioma advancement and novel therapeutic approaches for glioma.

## 2. Methods

### 2.1. Clinical Samples

We performed gene profiling of glioma patients from the Cancer Genome Atlas (TCGA) and healthy donors from the GTEx database by using the online website GEPIA (https://gepia2.cancer-pku.cn/#help). The expression of TMEM60 in tumor and nontumor tissues and the correlation between TMEM60 and GBM (glioblastoma multiforme) or LGG (brain lower grade glioma) prognosis were analyzed.

### 2.2. Cell Culture

Normal human brain astroglia cell line SVGP12, normal human astrocyte (HA), glioma cell line TJ905, GOS-3, U87MG, and SHG-44 were obtained from ATCC (Manassas, VA, USA). SVGP12 and U87 were cultured in EMEM (Hyclone, USA). HA was cultured in Astrocyte Medium (ScienCell, USA). GOS-3 and TJ905 were cultured in DMEM (Hyclone, USA). SHG-44 was cultured in RPMI 1640 (Hyclone, USA) [27]. All cells were cultured in a medium supplemented with 10% FBS (Gibco, USA) at 37°C incubation with 5% CO_2_.

### 2.3. Lentivirus Packaging and Infection

To generate the lentiviral shRNA constructs against human TMEM60, the TMEM60 shRNA sequences were cloned into the pLKO-puro vector. The sequences of shTMEM60 are as follows: shTMEM60-1, 5′-GAGTAACCCATGTAAATTACT-3′; shTMEM60-2, 5′-CGAGCTGGACTATCTGTGACT-3′. pLKO.1, pVSVG, pREV, and pGAG were cotransfected into HEK293T cells for 24 h, and cell culture media were collected. The full-length TMEM60 sequences were cloned into the pCDH-puro vector. pCDH, pSPAX.2, and pMD.2G were cotransfected into HEK293T cells for 24 h, and cell culture media were collected. The viruses were used to infect cells in the presence of polybrene. Forty-eight hours later, SHG-44 and U87MG cells were cultured in a medium containing puromycin for the selection of stable clones. The clones stably knocking down or overexpressing TMEM60 were identified and verified by western blotting [28].

### 2.4. Cell Viability and Apoptosis

Cell viability was determined by Cell Counting Kit-8 (CCK-8) assay and colony formation. For CCK-8 assay, cells were transfected with indicated oligonucleotides and seeded in 96-well plates at a density of 5,000 cells per well. After incubation for 24, 48, and 72 hours, 20 *μ*l CCK-8 (5 mg/ml) was added to each well, and the cells were incubated for another 4 hours. After that, the absorbance values at 450 nm were measured by using a microplate reader (Thermo, USA). For colony formation assay, the cells were suspended as single cells and seeded in 6-well plates (1,000 cells per well) and incubated for 10 days to form colonies [29]. The colonies were washed with PBS and dyed with 1% crystal violet for 20 minutes, captured, and counted. Cell apoptosis was evaluated by using the Annexin V/FITC Apoptosis Detection kit (Beyotime, China) as per the manufacturer's protocol. The cells were collected and detected on a flow cytometer (BD Biosciences, USA).

### 2.5. Western Blotting

The total proteins were extracted from cells after homogenization with RIPA lysis buffer (Beyotime), quantified by using a BCA assay kit (Beyotime). An equal amount of proteins was separated by SDS-PAGE, shifted to polyvinylidene fluoride (PVDF) membranes, and blocked with 5% skim milk in PBST for 2 hours, followed by incubation with primary antibodies against TMEM60, PARP, cleaved PARP, caspase-3, cleaved caspase-3, p-AKT, AKT, GSK3*β*, p-GSK3*β*, mTOR, p-mTOR, p70S6K, p-p70S6K, 4E-BP1, p-4E-BP1, and *β*-actin, at 4°C overnight. The next day, the protein bands were incubated with the corresponding horseradish peroxidase- (HRP-) coupled secondary antibodies, and enhanced chemiluminescence (ECL) visualization was performed on a gel image system (Bio-Rad) [30, 31].

### 2.6. Colony Formation

U87MG and SHG-44 cells were trypsinized, counted, and seeded in 6-well plates for 24 hours. Cells were cultured for 10 days to form visible clones. The clones were then washed, fixed, and stained with crystal violet, captured, and counted [32, 33].

### 2.7. Transwell Assay

The migration and invasion of glioma cells were determined by Transwell assay (Corning, USA). In brief, cells were placed into top chambers of 24-well plates with a serum-free medium, and the lower chambers were filled with complete medium [34]. After 48 hours incubation, the migrated cells were fixed with 4% paraformaldehyde (PFA) and then dyed with 1% crystal violet. For cell invasion, the upper chambers were coated with Matrigel (BD Biosciences, USA). The stained cells were observed and captured under a microscope [35].

### 2.8. Flow Cytometry

Flow cytometry was used to evaluate apoptosis of glioma cancer cells after TMEM60 knockdown. Glioma cancer cells were plated in 6-well plates with TMEM60 overexpression or vector as control. After double staining with fluorescein isothiocyanate- (FITC-) Annexin V and propidium iodide was performed using an FITC Annexin V Apoptosis Detection Kit (BD Biosciences) according to the manufacturer's recommendations [36], the cells were analyzed with a flow cytometer (FACScan; BD Biosciences) equipped with Cell Quest software (BD Biosciences). Cells were sorted into viable cells, dead cells, early apoptotic cells, and apoptotic cells, and the relative ratio of early apoptotic cells was compared with that of control cells in each experiment [37].

### 2.9. Statistics

Data in this study were presented as mean ± standard deviation (SD) of at least three independent experiments and processed by using the GraphPad software (USA). The student's *t* test or one-way analysis of variance (ANOVA) were conducted to compare differences between two or multiple groups. The *P* value <0.05 was considered statistically significant.

## 3. Results

### 3.1. The Expression of TMEM60 in Glioma Tissues and Cell Lines

We first identified the correlation between TMEM60 and glioma. The analysis on glioma patient samples and healthy donors from TCGA and the GTEx database showed that the levels of TMEM60 in glioma were remarkably elevated in GBM and LGC tumor tissues, compared with those in healthy tissues, and this elevated level of TMEM60 was correlated with poor overall survival of patients (Figures 1(a) and 1(b)). Moreover, the expression of TMEM60 was notably higher in glioma cell lines, including the TJ905, GOS-3, U87, and SHG-44, than that in normal human astrocyte cell lines (HA and SVG P12), as was manifested by mRNA and protein quantification (Figures 1(c) and 1(d)). These data suggested the abnormal upregulation of TMEM60 in glioma and its potential oncogenic role.

### 3.2. TMEM60 Facilitates Glioma Cell Proliferation

The abnormal overexpression of TMEM60 indicated that it may facilitate glioma progression [38]. To verify this speculation, we conducted stable knockdown or overexpression of TMEM60 in U87 and SHG-44 cells by infecting shRNAs (shTMEM60-1 and shTMEM60-2) or overexpressing vectors. The efficacy of infecting was determined by western blotting (Figures 2(a) and 2(b)). Results from CCK-8 indicated that TMEM60 knockdown alleviated cell viability in a time-dependent manner (Figure 2(c)), whereas the overexpression of TMEM60 facilitated cell viability (Figure 2(d)). Similarly, the decreased colony number in TMEM60-depleted GBM cells supported the proliferative role of TMEM60 in GBM (Figures 2(e) and 2(f)).

### 3.3. TMEM60 Promotes Glioma Cell Migration and Invasion

The high aggressiveness of glioma cells was also exhibited by cell migration and invasion [39]. Here, we performed Transwell assay to detect the metastatic ability of U87 and SHG-44 cells. As shown in Figures 3(a) and 3(b), knockdown of TMEM60 significantly suppressed the migrated and invaded glioma cells, and the histogram confirmed the statistical significance of the alteration (Figure 3(c)). By contrast, the overexpression of TMEM60 facilitated cell migration and invasion (Figures 3(d)–3(f)). These findings indicated that TMEM60 aggravated the aggressive phenotypes of glioma cells.

### 3.4. TMEM60 Suppresses Glioma Cell Apoptosis

After determination of cell proliferation and metastasis, we detected the apoptosis of U87 and SHG-44 cells [40]. As shown in Figures 4(a) and 4(b), the depletion of TMEM60 led to elevated apoptosis of glioma cells, as was manifested by the increased portion of early- and late-phase apoptotic cells. The detection of apoptosis-related signaling presented the emergence of cleaved PARP and caspase-3, along with the notable decrease of PARP and caspase-3 (Figures 4(c) and 4(d)). These results indicated that TMEM60 protects glioma cells from apoptosis.

### 3.5. TMEM60 Promotes the Glioma Cell Phenotype through PI3K/AKT Signaling

Studies have proved that the PI3K/AKT signaling contributed to aggressiveness of cancers, including glioma. Here in this work, we investigated whether TMEM60 modulates glioma cell behaviors through regulating the PI3K/AKT signaling pathway. Knockdown of TMEM60 suppressed the activation of PI3K/AKT signaling, as was manifested by decreased phosphorylation of Akt, GSK-3*β*, mTOR, p70-S6K, and 4E-BP1 (Figures 5(a) and 5(b)). Moreover, the overexpression of TMEM60 promoted the activation of PI3K/AKT signaling, as was manifested by increased phosphorylation of Akt, GSK-3*β*, mTOR, p70-S6K, and 4E-BP1 (Figures 5(c) and 5(d)). Therefore, TMEM60 promotes the hyperactivation of the PI3K/AKT signaling pathway in glioma cells.

## 4. Discussion

In the present work, we evaluated the role of a rarely reported gene TMEM60 in glioma carcinogenesis. We analyzed the expression of TMEM60 in patients with glioma and healthy donors and spotted its upregulation in glioma tissues compared with the nontumor tissues. The overall survival analysis also unraveled the correlation between high TMEM60 level with poor prognosis. It is well known that glioma is a highly aggressive malignancy with rapid proliferation [5]. Moreover, the glioma cells are capable of infiltrating to the neighboring brain tissues, causing pseudopalisading necrosis and angiogenesis, which consequently contribute to the poor prognosis of patients [17, 41, 42]. Other than the elevated level of TMEM60 in tumor tissues, we also found an elevation of TMEM60 in glioma cells compared with the normal human astrocyte cell lines.

To determine the specific role of TMEM60 in glioma carcinogenesis, we conducted knockdown and overexpression of TMEM60 in glioma cell lines and confirmed that TMEM60 overexpression led to enhanced cell viability, proliferation, migration, and invasion, as well as decreased cell apoptosis, which is consistent with the abnormal low level of TMEM60 in glioma tumor sections. Also, the knockdown of TMEM60 exerted opposite effects on GBM cell phenotypes. All these findings suggested that TMEM60 plays a potential oncogenic role in glioma [43, 44]. We next tried to decipher the mechanisms underlying the functions of TMEM60 during glioma carcinogenesis. Numerous studies have disclosed the high frequency of genetic aberrations in glioma, including the tumor protein p53 (TP53) [45, 46], cyclin-dependent kinase inhibitor 2A/B (CDKN2A/B) [47–49], tensin homolog (PTEN) [50, 51], EGFR [52, 53], PDGFRA [54], and PIK3CA, which leads to dysregulation of downstream signaling pathways such as the RB transcriptional corepressor 1 (RB1), PI3K/Akt/mTOR, and p53 [55–57]. The exploration of these genetic aberrations led to the discovery of targeted therapies against glioma [58–60]. PI3K/Akt/mTOR is a widely recognized signaling pathway that modulates the proliferation, motility, apoptosis, and angiogenesis in glioma [61–63].

Due to the abnormal cellular functions, elevated levels of PI3K and Akt are poor prognostic indicators for patients with malignancies [31, 64, 65]. Our study disclosed the alterations in the PI3K/Akt signaling under the overexpression or knockdown of TMEM60. Consistent with the prospected oncogenic role of TMEM60, TMEM60 overexpression upregulated the phosphorylation of PI3K/Akt signaling.

Taken together, we determined the aberrant expression of TMEM60 in glioma tissue samples and cell lines compared with the normal control. TMEM60 play an oncogenic role in glioma by promoting glioma cell proliferation, migration, and invasion and impairing cell apoptosis via activating the PI3K/Akt signaling pathway.

## Figures and Tables

**Figure 1:** TMEM60 expression in glioma. (a, b) Expression profile of TMEM60 in GBM and LGG from TCGA database was analyzed by the GEPIA website. T, tumor; N, nontumor adjacent tissue. (c, d) The transcription and protein expression of TMEM60 in human astrocyte cell lines, HA and SVG P12, and glioma cell lines, TJ905, GOS-3, U87, and SHG-44 by western blotting.

**Figure 2:** TMEM60 promotes glioma cell proliferation. U87 and SHG-44 cells were infected with shTMEM60 or negative control (shcon). (a) Western blotting experiment to detect the efficacy of shTMEM60 infection. (b) Western blotting to detect TMEM60 overexpression efficacy. (c, d) CCK8 assay was used to the proliferation of U87 and SHG-44 cells after infection of shTMEM60 or TMEM60 overexpression. (e, f) Colony formation assay was used for the proliferation of U87 and SHG-44 cells after infection of shTMEM60 or TMEM60 overexpression. The ratio of colony formation was quantified and calculated as histograms. All experiments were repeated independently for three times, and the representative one was shown. ^*∗∗*^*P* < 0.01 vs. shcon.

**Figure 3:** Effects of TMEM60 overexpression and knockdown on glioma migration and invasion. (a, b, c) U87 and SHG-44 cells of TMEM60 knockdown were examined for cell migration and invasion by Transwell assay. (d, e, f) U87 and SHG-44 cells of TMEM60 overexpression were examined for cell migration and invasion by Transwell assay. *N*=3, ^*∗*^*P* < 0.05, ^*∗∗*^*P* < 0.01 compared to the shcon or con group.

**Figure 4:** TMEM60 affects apoptosis of glioma cells. (a, b) Flow cytometry to detect U87 and SHG-44 cells' apoptosis alteration under the knockdown of TMEM60. The ratio of apoptotic cells was calculated and shown. (c, d) Western blotting assay to detect the expression of caspase-3, cleaved caspase-3, PARP, and cleaved PARP. All experiments were repeated independently three times, and the representative one was shown. ^*∗∗*^*P* < 0.01 vs. shcon.

**Figure 5:** The PI3K/AKT signaling pathway is involved in the effects of TMEM60. (a, b) The cell lysates were subjected to analysis of the phosphorylation levels of Akt and its downstream targets under the knockdown of TMEM60. (c, d) The cell lysates were subjected to the analysis of the phosphorylation levels of Akt and its downstream targets under the overexpression of TMEM60.

## Data Availability

The datasets used and/or analyzed during the current study are available from the corresponding author on reasonable request.

## Abbreviations

TCGA: The Cancer Genome Atlas
TMEM60: Transmembrane protein 60
PI3K: Phosphatidylinositol 3-kinase.
